This article has been retracted.

# A Decision Method for Benefit Distribution Mechanism of Shared End Distribution on Shapley Value

**DOI:** 10.1155/2022/3816440

**Published:** 2022-02-14

**Authors:** Hao Zhang, Yuan Hou, Feng-Feng He

**Affiliations:** ^1^Beijing Technology and Business University, Beijing Food Safety Research Base, Beijing, China; ^2^Beijing Technology and Business University, Beijing, China; ^3^Southwesten University of Finance and Economics, Chengdu, China

## Abstract

Online shopping has led to the rapid development of e-commerce, and at the same time, the pressure of offline distribution has increased abruptly. Therefore, a current development trend is to share end-to-end distribution against the background of the Internet. The main research content of this paper is the benefit distribution mechanism of shared end distribution. Based on an analysis of the current situation of interest distribution, this paper proposes factors that affect interest distribution from the perspectives of individuals and groups. The suitable income distribution mode of enterprise alliances is chosen from two dimensions—cooperation mode and coordination mechanism. Based on extant theory, this paper proposes a benefit distribution scheme-selection mechanism based on the modified Shapley value method and takes the terminal distribution in the Haidian District of Beijing as an example. The revised income distribution results better reflect the income-generating abilities of different enterprises within a cooperative organization and assign different benefit proportions to this cooperative organization based on different income-generating capacities to provide development incentives and, at the same time, better achieve income distribution.

## 1. Introduction

The terminal distribution cost of logistics enterprises remains constantly high; the key problem is that the dependence on human resources limits the ability of these enterprises to reduce human costs, and the allocation of logistics facilities resources is unreasonable [1–3]. The logic behind “Internet + logistics” is not applied to solve the problem of low-efficiency logistics operations. For example, cost waste is caused by an invalid operation caused by circuitous transportation, no-load transportation, and secondary distribution. To eliminate the dependence on human resources, improve the allocation efficiency of logistics facilities resources, and reduce the chances of invalid operations, it is necessary to make the end distribution operations automated, large-scale, systematic, and intelligent. Shared end distribution means that a number of logistics enterprises participate in the end distribution, that is, through connecting transfer points, order consolidation, and other ways to integrate end distribution infrastructure resources to provide low-cost and efficient end distribution services [4, 5]. Shared end distribution through horizontal logistics integration, that is, the unified scheduling of the resources of many logistics enterprises, is carried out to realize the scale and intensification of regional end distribution operations and to better adapt to the current economic development situation from the two aspects of efficiency and effectiveness so as to achieve low-cost and high-efficiency end distribution services. The joint distribution mode, which takes the logistics enterprise as the hub and connects the e-commerce platform with the logistics terminal distribution service, is the solution to the bottleneck problem encountered by the current e-commerce platform in the terminal distribution link. As the sharing mode of the third-party collection platform expands in the form of joining, it is difficult to standardize and standardize the work in this process. The joint distribution model participates in a variety of enterprise levels, which is not conducive to the coordination between enterprises and the integration of resources. The intelligent express cabinet sharing mode takes the intelligent express cabinet as the carrier to connect the terminal logistics service and users; on the one hand, it saves the increase in operating costs caused by decentralized business outlets, and on the other hand, it uses mobile Internet technology to integrate offline physical resources and collect online service data, which not only reduces costs and increases efficiency but also simplifies the traditional terminal distribution service process and improves the quality of terminal distribution service. Let the terminal distribution service realize digitalization, informationization, and intellectualization.

When constructing the alliance of shared end distribution logistics enterprises, we have to consider the size of each enterprise, the core competitiveness, and the logistics demand of each region. Is it possible to build alliances among enterprises of different sizes? If so, what principles do you need to follow to build an alliance? In the formation of the enterprise alliance, how to protect the core competitiveness of the enterprise itself without affecting the interests of the whole enterprise alliance? In addition, what factors will hinder or promote the establishment and stability of logistics enterprise alliance? Answering the above questions is of great significance for building a shared terminal distribution platform for logistics enterprises. The main research of this paper is aimed at studying the cost-sharing ratio of each enterprise from the perspective of resource utilization efficiency, and most of the literature focuses on improving this ratio by increasing the risk factor or effort level on the basis of the Shapley value method. From the perspective of the sharing economy, this paper studies the impact of enterprises on cost allocation due to resource utilization efficiency from the point of view of the better promotion of resource integration.

## 2. Literature Review

### 2.1. Research Status of Shared End Distribution

Against the background of “Internet + logistics,” sharing economy thinking is applied to the logistics industry, which continuously releases the resource dividend of integrated logistics. For the “theme of shared terminal distribution,” scholars have mainly focused on the following three aspects: site selection for terminal distribution outlets, the optimization of terminal distribution path, and research on sharing terminal distribution mode. Perez-Mesa et al. [6] established a location selection model for FMCG's agricultural product distribution center with the lowest total cost. Zhang and Liu [7] proposed the method of a gray demand logistics distribution center location and model of a gray sales demand logistics distribution center location planning, which can solve the problem of gray sales demand in logistics distribution center location. Kexin et al. [8] adopted the node centrality index of complex network theory to evaluate the importance of existing terminal distribution outlets. Evari et al. [9] found that using friends in a social network to assist in last-mile delivery greatly reduces delivery costs and total emissions while ensuring speedy and reliable delivery. In addition, Li et al. [10] analyzed the ability of logistics enterprises to meet the diversified needs of service objects through the differentiation of asset allocation. Moreover, Yu et al. [11] believed that the application of the ant colony algorithm has good feasibility for the distribution path optimization of logistics terminals. Tang et al. [12] solved the model based on multiphase particle swarm optimization algorithm (MPPSO) and Matlab. Masoud et al. [13] applied a genetic algorithm and hybrid genetic algorithm to calculate path optimization schemes and compared the results. At present, genetic algorithms are more commonly used to solve this type of problem [14–17].

Studies on the theme of the shared terminal distribution mode mainly include the following. Patterson et al. [18] established a carrier selection model, the results of which show that third-party logistics are more dependent on multimodal transport than are other terminal carriers. Lu et al. [19] applied the routing optimization algorithm to establish a multiagent simulation model to solve the routing optimization problem for electric vehicles. In the context of “Internet plus Internet of Things,” Ryu et al. [20] proposed an integrated semantic service platform to support ontological models in various IoT-based service domains of a smart city. The driving factors for the formation of end-to-end joint distribution alliance are as follows. First, to meet the needs of e-commerce economic development, with the increasing maturity of e-commerce, with the upgrading of consumption, the end distribution business shows a substantial growth, and the traditional end distribution model can no longer adapt to large-scale offline distribution business [21]. The second is the need to reduce the cost structure. On the one hand, because of the high intensity of work and low wages, the mobility of end distribution employees is extremely high, and the human cost of end distribution remains high. On the other hand, the scale of operation and market limits the ability of a single enterprise to integrate resources. Third, the need to improve the efficiency of distribution. Due to the large number of service objects and the scattered geographical location, express delivery enterprises usually increase the distribution cost because of unreasonable distribution routes, high load rate, secondary distribution, and other problems [22]. Fourth, the needs of high-quality end distribution services; end distribution services gradually show a face trend, that is, with user experience as the core, personalized end distribution services are provided based on user portraits through big data, artificial intelligence, and other technologies. Fifth, to advocate the need of green logistics, the establishment of end-to-end joint distribution alliance is conducive for the integration of logistics infrastructure and other resources, and for reasonable planning of vehicle transport routes, so as to reduce traffic pollution and achieve energy saving and emission reduction.

### 2.2. Research Status of the Benefit Distribution of Logistics Alliances

Releasing the dividend of logistics integration enables end distribution enterprises to reduce costs and increase efficiency. The design and operation of logistics alliances are critical, especially the distribution of benefits. The current research in this field is mainly classified as below.

Based on the Shapley value method and modified to put forward a benefit distribution strategy, an increasing number of scholars have used the Shapley value method to conduct benefit distribution research [23, 24]. Gong et al. [25] examine the production coordination problem from the perspective of asymmetric information. Wei [26] constructed a Shapley value model of income distribution in the information flow of a construction supply chain under asymmetric information to ensure the security of the synchronous control of information flow and a more balanced benefit distribution. Pan and Fang [27] established an integrated energy service benefit distribution model based on the improved Shapley value method to break the imbalance between the environment and economy of integrated energy services to realize overall sustainable development. Improving the Shapley value method can reduce the economic loss caused by downtime and promote multi-factory cooperation [28]. In addition, through the application of the improved Shapley value method, the production and delivery time cycle will be shortened and found that it can be applied to any industry of concern to improve operations [29].

There are many studies on the distribution of multiagent interests, and the methods used are very diverse. Lian [30] through constructing a fuzzy time window-based scheduling optimization model for the cross-docking of cold chain logistics found that the distribution time of cold chain logistics can be significantly shortened and the distribution cost, damage cost, and economic benefits can be significantly reduced. Ma et al. [31] established a cold chain dynamic game model involving a milk manufacturer and two downstream oligopoly supermarkets under a wholesale price contract. Sun et al. [32] proposed a two-layer programming model to find the optimal location of a logistics distribution center by considering the advantages of customers and logistics planning departments. Some scholars have used the benefit distribution model of coastal port intelligent logistics supply chains based on intelligent bionic swarm evolution optimization control [33–35] or the profit distribution model based on agents [36–38] to realize the benefit distribution among multiple agents. Nadia et al. [39] through investigation and analysis proposed the necessity and importance of establishing alliances for enterprises and analyzed the interests of an alliance as a whole by using the Shapley value method. Meng et al. [40] studied multiorganization cooperation under the sharing economy model, which provided a theoretical basis for core enterprises to formulate reasonable income distribution strategies and promote the sustainable development of the sharing economy. Shang et al. [41] adopted cooperative game theory and the Shapley value method to solve the benefit distribution scheme, which improved overall risk management ability and business stability and stimulated the development potential of the enterprise.

On the whole, scholars focus on the macro research and analysis of the mode construction of shared end distribution, and pay more attention to the path optimization and site selection in shared end distribution on the micro level, but rarely analyze and study the problems in the practice of shared end distribution from the perspective of enterprise cooperation. How to complete the terminal distribution operation with the lowest cost, the least manpower, and the highest efficiency is the main problem that express delivery enterprises are facing. At present, the repeated construction of business outlets leads to the waste of social resources, the recruitment difficulties of grass-roots express salesmen, and the secondary distribution caused by the timeliness of information, making the “lone Wolf” tactic easy to suffer losses in the terminal distribution service, so it is imperative to jointly build and share logistics. It is very important to design a fair and reasonable benefit distribution mechanism to realize the sustainable development of sharing terminal distribution alliance.

## 3. Research on the Benefit Distribution Mechanism of Shared End Distribution

This paper investigates the factors that affect the benefit distribution of enterprises from the perspective of groups and individuals, as shown in Table 1, and gives the income distribution model of shared end distribution, as shown in Table 2, as follows:

When rational people participate in games involving economic activities, the two problems that need to be solved are that related to cooperation and that related to coordination. The cooperation mode is defined as the negotiating and signing of agreements to define the responsibilities and obligations of participants, and the coordination mechanism to achieve stable income expectations through good institutional design provides incentives and signals for all parties to maintain cooperation loyalty. Different cooperation modes mean that cooperative organizations have different degrees of alliance cohesion, and coordination mechanisms with different stable income expectations have different incentives and signals for members to provide cooperation. In addition, because the problems of cooperation and coordination are the two sides of game behavior, respectively, a certain cooperation model is bound to correspond to a coordination mechanism. As shown in Figure 1, the cooperation type of outsourcing business in the form of a market contract corresponds to the fixed wage model that allows for payment for a certain volume of business according to the settlement scheme; the strategic alliance model that aims to dilute the enterprise boundary to realize the sharing of management rights corresponds to the payment mode of land rent based on the distribution of alliance income on the basis of fixed payment. The ecological competition type with Internet technology as the background corresponds to the shared profit model, which is based on the coconstruction and sharing of logistics infrastructure and information resources as well as the benefits of the alliance.

## 4. The Benefit Distribution Scheme of the Modified Shapley Value Method

The Shapley value method is proposed by L. S. Shapley to solve the n-person cooperative game problem. The application of this mathematical algorithm to the benefit distribution of alliance members can effectively avoid egalitarianism in distribution. The contribution ability of the members of the cooperative organization is included in the income distribution, which effectively arouses the production enthusiasm of the members. If *n* individuals participate in a social and economic activity, when the cooperative nature of the parties is greater than the competitive nature, the parties can obtain higher benefits by forming a cooperative relationship than under the conditions of individual operation, and with the increase of the scale of the cooperative organization, the industrial synergy effect based on resource sharing and information exchange will become more prominent, and the income of the cooperative organization will gradually increase. A reasonable distribution scheme will provide corresponding organizational incentives to the members of the cooperative organization, and then ultimately ensure that the interests of all n-person cooperation can be maximized.

### 4.1. Shapley Value Method Based on Contribution Degree Distribution

For *f* a weighted voting scheme used by *n* voters to choose between two candidates, the *n* Shapley-Shubik Indices (or Shapley values) of *f* measure how much control each voter can exert over the overall outcome [42]. Suppose that there are *n* individuals participating in cooperation, and all participating members are denoted by *N* = {1,2, ....., *n*}; any subset *S* of *N* (any cooperative combination in n-person cooperation) has a corresponding real-value function *V* (S), that is, the benefits that can be obtained by any cooperative combination S. *V* (*φ*) = 0, which means that if there are no participants in the cooperative organization, then the total income of the alliance is 0. Suppose that *S*_1_ and *S*_2_ are any two kinds of cooperative combinations in N and satisfy *S*_1_∩*S*_2_ = ∅. The profit created by an alliance formed by these two combinations is greater than the sum of the profits generated by these two combinations; that is, *V* (*S*_1_∪*S*_2_) > *V* (*S*_1_) + *V* (*S*_2_). Thus, [*N*, *V*] is called the n-person cooperation strategy set. In a set of allocation strategies, it is assumed that *X*_i_ indicates that the maximum income *V* (*N*) obtained by member *N*_i_ in the alliance is a share of income, that is, the Shapley value, and the distribution strategy set of the alliance in the cooperative game is represented by *X* = {*X*_1_, *X*_2_ ....., *X*_*n*_}. The distribution set should meet two basic constraints—overall and individual rationality. That is, the sum of the benefits of the alliance as a whole is equal to the sum of the benefits of each member, and the income of individual members in the alliance is greater than that of individual members who complete the task alone, which is expressed by the following mathematical formula:

(1) $$\begin{array}{c} \text{overall rationality}:\sum_{i=1}^{n}xi=V\left(N\right),\\ \text{Integrated rationality}:X\left(i\right)>V\left(i\right). \end{array}$$

According to the basic theorem of the Shapley value method, in the cooperative organization of *n* people, under characteristic function *V*, the income of each member is expressed by *X* = {*X*_1_, *X*_2_ ......., *X*_*n*_}. According to the Shapley value method, the income of each member can be obtained as follows:

(2) $$\begin{array}{c} X_{i}=\sum_{s\in Si}W\left|S\right|\left[V\left(S\right)-V\left(S-i\right)\right]. \end{array}$$

The formula explains the following:

1. |*S*| represents the size of the organization
2. *W*(|*S*|) is a weighting factor, *W*(|*S*|)=((*s*) − 1!(*n* − |*S*|)!/*n*!).
3. *V*(*S* − *i*) represents the benefits of the organization when member *i* is removed from organizational alliance S
4. *V*(*S*) − *V*(*S* − *i*)  represents the contribution made by member *i* in the organizational alliance.

According to the above introduction to the Shapley value method, we know that this method takes the contribution of each member as the distribution standard in the benefit distribution, and the premise behind this distribution method being considered reasonable and fair is that the members of the organizational alliance conform to the rational person hypothesis, and the costs and risks borne within the organizational alliance are consistent. However, compared with the specific practice, due to the differences between enterprise qualification and the competitive environment, there is a gap between the cost and risk shared by enterprises with different strengths in the organizational alliance because of the differences in their competitiveness. This kind of risk and cost gap can be shown through the cooperation mode and income distribution mechanism in the organizational alliance. When calculating members' income by the Shapley value method, it is assumed that members' ability to share the cost is consistent with the risk, which leads to the final calculation result of the Shapley value method deviating from the facts and being unable to provide the corresponding compensation mechanism for those enterprises that bear high costs and risks. Therefore, this paper hopes to modify the results calculated by the Shapley value method by measuring the evaluation indicators of different cooperation modes and income distribution mechanisms and forming weighted factors to obtain a more reasonable benefit distribution scheme that takes into account the costs and risks borne by enterprises in the cooperative organization.

### 4.2. Revision of the Shapley Value Method and Establishment of the Model

In this paper, the evaluation standard of enterprises under an established cooperation mode is based on the influencing factors of benefit distribution from the perspective of groups and evaluates the influencing factor Ai of an enterprise on organizational income output under this cooperation system from three aspects: the strength and status of alliance members, the unit price and market demand of services, and the stability of the logistics alliance relationship. The cooperation mode of sharing resources explores the influencing factors of interest distribution at the macro level of cooperative organizations, while the coordination mechanism of income distribution explores those at the micro level of alliance members. From the perspective of individual enterprises, the influencing factors of benefit distribution mainly have the following four levels: cost input, risk taking, service level, and marginal contribution. The correction results for the two angles are shown in Tables 3 and 4.

The influencing factors of the three cooperation modes on the income distribution strategy are expressed by *A*_j_ = {*A*_1_, *A*_2_, *A*_3_}, and the following conditions are met:

−1<*A*_*i*_<1; −1<*a*_ij_<1
2. ∑_*j*=1_^3^*aij*=1
3. ∑_*j*=1_^3^*Aj*=0

The influencing factors of the three income distribution coordination mechanisms on the income distribution strategy are expressed by *B*_*j*_ = {*B*1, *B*2, *B*3}, and the following conditions are met:

−1<*B*_i_ < 1; −1<*b*_ij_<1
2. ∑_*j*=1_^3^*bij*=1
3. ∑_*j*=1_^3^*Bj*=0

### 4.3. Establishment of the Modified Shapley Value Model

The Shapley value has become popular in the Explainable AI (XAI) literature, thanks, to a large extent, to a solid theoretical foundation, including four “favourable and fair” axioms for attribution in transferable utility games. The Shapley value is probably the only solution concept satisfying these axioms [43]. From the overall rational point of view, this paper probes into correction factor *A*_*i*_ of each enterprise in three aspects: the strength and status of alliance members, the unit price of service and market demand, and the stability of logistics alliance relationships from a group perspective. Yokote [44] introduced a new axiom, called equilibrium contribution property of equal contributors, and proved that this axiom characterizes a new class of solutions together with validity and weak covariance, providing a new axiom basis for analyzing variations of Shapley values in a uniform way. Brin [45] proved that the Shapley value is characterized by this fairness, efficiency, and the nature of the person in the empty game, and these three axioms also characterize the Shapley value of a simple game class. From the perspective of individual rationality, this paper studies the correction factor *B*_*i*_ of enterprises under the four dimensions of cost input, risk taking, service level, and marginal sharing. To make the final quantitative results more in line with the specific situation in practice, the evaluation indicators of all levels and dimensions are divided into different weights, thus reflecting the unequal impact of various factors on the final benefit distribution scheme [46, 47]. After quantification, we obtain correction factor *A*_i_ of each enterprise under overall rationality and the correction factor of individual rationality *B*_*i*_. By taking the average of both, we finally obtain the comprehensive correction factor of each enterprise, that is, 1/2^*∗*^ (*A*_i_ + *B*_i_). Through the comprehensive correction factor calculation, we can obtain the correction value that should be obtained by each enterprise and finally obtain the benefit distribution scheme.

In a cooperative organization of *n* people, under characteristic function *V*, the benefit of each member is expressed by *X* = {*X*_1_, *X*_2_......, *X*_n_}. Taking the Shapley value as the basic original value *X*_i_, the cooperative income distribution strategy is modified from the two aspects of the cooperation mode of shared resources and the coordination mechanism of income distribution; correction factor 1/2^*∗*^ (*A*_i_ + *B*_i_) is obtained; and correction value △*X*_i_, Δ*Xi*=(1/2) × *Xi* × (*Ai*+*Bi*) is obtained. The income of each member after the amendment is expressed by *X*′={*X*_1_′, *X*_2_′,…, *X*_*n*_′}, *X*_*i*_′(*V*)=*X*_*i*_(*V*)+Δ*X*_*i*_(*V*). The specific correction process is shown in Figure 2.

## 5. Example Analysis

### 5.1. Enterprise End-to-End Distribution Costs

Bi et al. [48] conducted an empirical study on five express delivery enterprises in China and made a comparative analysis of the results. Li [49] analyzed the problems existing in logistics distribution of express delivery enterprises, discussed various factors affecting customer satisfaction, and put forward empirical analysis assumptions. So the example analysis of this paper selects express delivery enterprises under joint distribution as the research objects and applies the correction method to modify the initial Shapley value based on the Shapley value method to obtain a more realistic distribution scheme. This paper takes 10 distribution outlets of Yuantong, Zhongtong, and Best Express enterprises in Haidian District as the research objects and studies the distribution costs borne by each enterprise under three forms of distribution: three enterprises participate in the distribution task alone; two enterprises cooperate to participate in the joint distribution, and another enterprise participates in the distribution alone; and three enterprises cooperate to participate in the joint distribution. The corresponding distribution outlets and their numbers are shown in Table 5.

#### 5.1.1. Three Enterprises Participate in Distribution Separately

The scheme and cost for the three enterprises to participate in distribution separately is shown in Table 6:

#### 5.1.2. Two Enterprises Cooperate to Participate in Distribution

A. Yuantong cooperates with Zhongtong to participate in distribution, and Yunda distributes separately, the distribution path and cost are shown in Table 7:

B. Yuantong and Yunda cooperate to participate in distribution, and Zhongtong distributes separately, the distribution path and cost are shown in Table 8:

C. Yunda cooperates with Zhongtong to participate in distribution, and Yunda distributes separately, the distribution path and cost are shown in Table 9:

#### 5.1.3. Three Enterprises Participate in Joint Distribution

The distribution cost under the cooperation of the three enterprises is shown in Table 10:

### 5.2. Distribution of Alliance Income by the Shapley Value Method

By calculating the costs of distribution schemes under the above cooperation modes, we can obtain the costs shared by enterprises in different distribution schemes and the benefits generated by joint distribution. On this basis, the initial Shapley values of the three enterprises after forming a cooperative organization can be calculated. To facilitate the latter description, Yuantong, Zhongtong, and Yunda enterprises are replaced by enterprises 1, 2, and 3, respectively.

As can be seen from Table 11, the participation of enterprises in joint distribution can effectively help them generate organizational cooperation income, with all three companies undertaking distribution tasks alone as the lowest threshold. When the number of enterprises participating in joint distribution continues to increase, the overall cooperation income increases significantly. In the example analysis of this paper, the total cost of the three enterprises participating in the distribution alone is 285.95. However, when the two enterprises cooperate, they obtain the benefits of the cooperative organization relative to the other enterprise that does not participate in the cooperation. Cooperation between Yuantong and Zhongtong can generate 91.1 units of income, and that between Yuantong and Yunda enterprises can generate 106.15 units of income. Moreover, cooperation between Zhongtong and Yunda enterprises can produce 89.2 units of benefits. From the perspective of bilateral cooperation, the profits of enterprises are better when they cooperate with stronger enterprises. The income from cooperation among Yuantong, Zhongtong, and Yunda is higher than that between Zhongtong and Yunda. From the perspective of multilateral cooperation, with the increase in the number of cooperative enterprises, the income of cooperative organizations also significantly increases. When the three enterprises work together to participate in a joint distribution, the terminal distribution cost can be significantly reduced by 60.6%. As a result, the profit ceiling of each enterprise at the end of distribution is raised. As large logistics enterprises gradually complete the primitive accumulation of enterprise development, gradually move toward the intelligent logistics mode in the unmanned era, and eliminate the dependence on human resources, small and medium-sized logistics enterprises, due to limited funds and a lack of technology, on the one hand, cannot realize the reform of operation mode in a short period of time. On the other hand, if enterprises continue to follow the traditional logistics management model, then they still face the constraints of human costs, so the living space of small and medium-sized logistics enterprises is gradually narrowed. In this paper, through an analysis of examples, we know that when small and medium-sized enterprises are facing strong competitors such as large logistics enterprises, if they want to overtake them, then the establishment of a cooperative cooperation model and benefit distribution coordination mechanism suitable for the development of enterprises is necessary for their long-term development.

According to the above model of the Shapley value method and combined with the research object in the example analysis, we know that our research objects are three express delivery enterprises, namely, enterprises 1, 2, and 3, represented by the set *N* = {1, 2, 2, 3}. The income earned by each enterprise in the cooperative organization is expressed by *X* = {*X*_1_, *X*_2_, *X*_3_}. The calculation process and results are shown in Tables 12–14.

According to the above calculations, under the Shapley value model, the income of each enterprise participating in the joint distribution is as follows:

(3) $$\begin{array}{c} X_{1}=15.19+17.7+28.98=61.86,\\ X_{2}=15.19+14.87+23.33=53.39,\\ X_{3}=17.7+14.87+28.35=60.91. \end{array}$$

In the distribution scheme of the Shapley value model, there is little difference in the organizational income of the enterprises participating in the joint distribution, which stems from the assumption at the beginning of the establishment of the model: the differences among participants should be ignored. However, due to the different qualifications of each enterprise, the contribution ability of the heterogeneous enterprise resources to the cooperative organization is different. When the heterogeneous enterprise resources help the cooperative organization achieve high returns, this part of the income should be compensated to the enterprise in terms of contribution ability to provide the cooperative organization with the development incentive of “contributing enterprise resources.” Only in this way can the sustainable and coordinated development of the cooperative organization be realized.

### 5.3. Modification of the Initial Shapley Value

The following is the correction of the initial Shapley value of each enterprise obtained through the example analysis. The source of the correction factor is based on the evaluation indicators of each enterprise in three aspects: the strength and status of alliance members, service unit price and market demand, and the stability of the logistics alliance relationship. The feedback source of the evaluation index of the enterprise is mainly obtained by network enterprise data and offline interviews and quantifies the evaluation index of each enterprise according to first-hand data.

The initial Shapley value of the enterprise is modified from the point of view of the cooperation mode of sharing resources, and the details of the correction factors of each enterprise are shown in Table 15.

The initial Shapley value of the enterprise is modified from the point of view of the coordination mechanism of income distribution, and the correction factors of each enterprise are shown in Table 16.

Through the above calculations, the final benefit distribution correction factors of the three enterprises participating in joint distribution can be obtained. To make the correction results more reasonable by averaging the correction factors from two perspectives, by calculating the final correction factors of each enterprise, correction value △*Xi*, △*Xi* = *Xi*^*∗*^1/2 (*Aj* + *Bj*) is finally obtained. The specific results are shown in Table 17.

Yuantong Express is ahead of the other two enterprises in terms of overall market share and service quality, and its business orders are also greater in amount and number than are those of the other two enterprises, which will make an important contribution to the income of the whole cooperative organization in the process of building the alliance. Yunda Express has weak market share and resource scheduling ability compared with Yuantong and Zhongtong enterprises, showing positive externalities to organizational income. With the help of cooperative organizations, the Yunda enterprise reduces the cost of terminal distribution and obtains the opportunity to share the benefits from cooperation, but to compensate for the contribution of Yuantong and Zhongtong, part of its income needs to be allocated to them to send a positive incentive signal to them in terms of contribution. Therefore, by observing the correction factors of various enterprises, we can see that those of the Yuantong and Zhongtong enterprises are positive, while the correction factor of the Yunda enterprise is negative. Since the main purpose of this step is to calculate the correction value of each enterprise, the correction value further modifies the distribution scheme on the basis of that obtained by the Shapley value method, so the sum of the correction value of each enterprise should be equal to 0; that is, the correction scheme of the paper does not change the income of the cooperative organization in the whole correction process. On the basis of this modified value, we can obtain the final distribution scheme by adding the initial Shapley value calculated by the Shapley value method, and the final distribution scheme is compared with that obtained by the Shapley method, as shown in Table 18:

Through the above comparison, we can see that the distribution scheme of the Shapley value method pays more attention to the distribution of cooperative income from the perspective of average distribution, and there is little difference in the respective income of the three enterprises. This “average” distribution method does not give compensation and incentives to the contribution ability of enterprises with different qualifications, which is not conducive for the sustainable development of cooperative organizations. In the example analysis of this paper, we can see that based on the distribution scheme according to the Shapley value method, the cooperative benefits shared by the three enterprises are not very different, and the difference is controlled within 9 units. The distribution scheme under the average principle cannot reflect the utility of each individual in the cooperative organization, quantify this utility, and reward this utility through reasonable benefit compensation. In the example analysis of this paper, the Yuantong enterprise can bring higher business order and resource scheduling ability to the cooperative organization and can share its offline logistics resources with other enterprises; after revision, the income of the Yuantong enterprise is obviously higher than that of the Zhongtong and Yunda enterprises.

The case study of this paper takes joint distribution as the research background, so in general enterprise practice, we usually choose the cooperation mode of diluting enterprise boundary, which is higher than outsourcing cooperation. The core of collaborative joint distribution is sharing orders. When strong enterprises share internal low-profit orders with members of cooperative organizations, while other members complete these orders to harvest enterprise profits, it is necessary to pay a corresponding proportion of “rent” to stronger enterprises, which is also the basic idea of the mode of paying land rent in the coordination mechanism of income distribution. This kind of “rent” incentive is to make stronger enterprises more willing to participate in the construction of cooperative organizations, so as to maintain the sustainable development of cooperative organizations. In this case, because of its limited market share and service level, Yunda enterprise undertakes the terminal distribution business of high cost and low volume when it operates alone. However, when the distribution business is optimized through joint distribution, from its own vertical comparison, Yunda enterprise not only completes the corresponding distribution tasks but also obtains the benefits of cooperation. However, the stability of this form of cooperation depends on the comparison of the strength of their respective enterprises, which is mainly reflected in the market share; comprehensive service capacity; and complete infrastructure. In terms of logistics resource scheduling ability, when the strength of enterprises is very different and the balance of cooperation is broken, enterprises with greater discourse power will force weaker enterprises to accept organizational agreements that are not conducive for the development of enterprises, which is likely to break the calm mode of cooperation.

## 6. Conclusions

This paper focuses on the difficult problem of enterprise cooperative benefit distribution in end distribution, takes the benefit distribution principle as the basic constraint, and constructs a two-dimensional enterprise evaluation system from the group and individual perspectives. The income distribution mode selection matrix is constructed from the two dimensions of the cooperation mode and coordination mechanism. Under these different practical backgrounds, all enterprise parties choose the appropriate cooperation mode and income distribution mode in the income distribution mode selection matrix and obtain the income distribution correction factor from the evaluation system within the selected range, which is modified on the basis of the initial Shapley value. Compared with the initial Shapley value method, which pursues income equalization, the revised income distribution results more so reflect the income-generating ability of different enterprises in the cooperative organization and give different proportions of benefits to the cooperative organization based on different income-generating capacities to provide incentives for the development of the cooperative organization. This paper holds that the influence of the income distribution scheme of cooperative organizations depends on the close relationship between the cooperation mode of shared resources and the coordination mechanism of income distribution. Under this two-dimensional mechanism, the final benefit distribution should be determined based on the evaluation of the enterprise and not on only the Shapley value mathematical model. The two-dimensional selection mechanism based on income distribution can better reflect the income-generating ability that enterprises can exert in the specific cooperation practice. From a rational point of view, this paper proposes what kind of cooperation mode and coordination mechanism enterprises should be established to realize the sustainable development of cooperative organizations. However, in practice, it is still necessary to make prudent cooperation decisions based on an enterprise's internal resources, enterprise strategy, enterprise organizational structure, and the external environment.

This paper focuses on studying and solving the problem of the benefit distribution of various enterprises, puts forward a framework solution from the perspective of static research, and presents a two-dimensional selection matrix of income distribution based on overall and individual rationality. The Shapley value algorithm is modified from the point of view of the cooperation mode and income distribution coordination mechanism. Although this paper takes into account the influencing factors of overall rationality on income distribution and individual rationality on income distribution, it does not specifically analyze the influence of the negotiation premium power between different enterprises on the whole income distribution, that is, taking into account the rationality of the establishment of cooperative organizations and the rationality of individual participation in cooperative organizations, but there is no dynamic research perspective for analyzing the continuous growth of enterprises in cooperative organizations. Whether the old cooperation model and distribution mechanism can still be established needs to be further studied. Therefore, this paper does not consider the dynamic cooperative development of enterprises, and the static research perspective on the distribution of interests of enterprises inevitably makes the final research results deviate from the practices of specific enterprises.

## Figures and Tables

**Figure 1:** Income distribution mode selection matrix.

**Figure 2:** Modification process of the Shapley value method.

**Table 1:** Influencing factors of enterprise benefit distribution in end-to-end distribution.

	Influencing factors	Meaning
Group.Visual angle	Strength and status	It determines the size of the bargaining chips of the members in the distribution of interests
	Service unit price and demand	It determines the bottom line in terms of cost that the enterprise alliance can bear and the ceiling of profit expectation
	Alliance stability	It determines whether the alliance cooperation relationship is long term or short term

Individual.Visual angle	Cost input	It determines the proportion of benefit distribution among participants
	Risk bearing	It can be divided into external and internal risk
	Service level	It determines user satisfaction
	Marginal contribution	The higher the marginal contribution rate is, the higher the sovereign status in the distribution of interests

**Table 2:** Income distribution model of shared end distribution.

	Income distribution model	Concrete
Cooperation mode of sharing resources	Outsourcing collaboration	Outsourcing of noncore logistics business
	Strategic alliance type	Dilution of enterprise boundaries through organizational cooperation agreements
	Ecological competition and cooperation	Drawing of lessons from the social organization of human beings and the operating mechanism of natural ecosystem

Coordination mechanism of income distribution	Fixed wage model	Expected coordination mechanism in the environment of outsourcing collaboration
	Mode of paying land rent	Specific monetary quantification of the benefits from resource acquisition
	Shared profit model	Emphasize that all parties should participate in the construction of logistics infrastructure and share the benefits of such cooperation

**Table 3:** Enterprise evaluation system from a group perspective.

Influencing factors of benefit distribution from a group perspective	Weight	Enterprise 1	Enterprise 2	Enterprise 3
Strength and status of the members of the alliance	0.5	*a*_11_	*a*_21_	*a*_31_
Service unit price and market demand	0.3	*a*_12_	*a*_22_	*a*_32_
Stability of the logistics alliance	0.2	*a*_13_	*a*_23_	*a*_33_
Correction factor of enterprise i	—	*A*_1_	*A*_2_	*A*_3_

**Table 4:** Enterprise evaluation system from an individual perspective.

Influencing factors of benefit distribution from an individual perspective	Weight	Enterprise 1	Enterprise 2	Enterprise 3
Cost input	0.3	*b*_11_	*b*_21_	*b*_31_
Risk bearing	0.3	*b*_12_	*b*_22_	*b*_32_
Service level	0.3	*b*_13_	*b*_23_	*b*_33_
Marginal contribution	0.1	*b*_14_	*b*_24_	*b*_34_
Correction factor of enterprise i	—	*B*_1_	*B*_2_	*B*_3_

**Table 5:** Distribution outlets and corresponding numbers.

Serial number	1	2	3	4	5
Distribution network	Yongfeng 1	China Agricultural University 2	Space bridge 3	Learn to clear the way 4	Beijing University of Aeronautics and astronautics 5
Serial number	6	7	8	9	10
Distribution network	Tsinghua university 6	Shangdi 7	Xiangshan 8	Zhongguancun 9	Longevity road 10

**Table 6:** Distribution costs of individual operations in enterprises.

Each enterprise distributes separately	Distribution route	Mileage	Traffic demand	Call vehicle	Loading rate (%)	Distribution cost
Yuantong	0-4-2-6-9-0	42.2	423.30	3	84.66	103.7
	0-7-1-0	40.5	179.31		35.86	
	0-5-3-8-10–0	64.7	441.70		88.34	
Zhongtong	0-2-1-7-0	30.3	261.25	3	52.25	86.65
	0-6-5-9-0	17.7	249.90		49.98	
	0-4-3-8-10–0	65.3	332.15		66.43	
Yunda	0-5-4-6-0	25.9	274.16	3	54.83	95.6
	0-3-2-9-7-0	46.5	325.64		65.13	
	0-10-8-1-0	58.8	260.52		52.10	

**Table 7:** Distribution costs under cooperation between Yuantong and Zhongtong

Yuantong-Zhongtong joint distribution	Distribution route	Mileage	Traffic demand	Transfer vehicle	Loading rate (%)	Distribution cost
Yuantong	0-4-5-6-9-7-0	47.5	964.38	2	96.44	43.75
Zhongtong	0-2-10-3-8-1-0	71	835.97	2	85.40	55.5
Yunda	0-5-4-6-0	25.9	274.16	3	54.83	95.6
	0-3-2-9-7-0	46.5	325.64		65.13	
	0-10-8-1-0	58.8	260.52		52.10	

**Table 8:** Distribution costs under cooperation between Yuantong and Yunda.

Yuantong-Yunda joint distribution	Distribution route	Mileage	Traffic demand	Transfer vehicle	Loading rate (%)	Distribution cost
Yuantong	0-4-2-6-5-9-0	40.5	939.94	2	93.99	40.25
Yunda	0-3-8-10-7-1-0	65.8	964.69	2	96.47	52.9
Zhongtong	0-2-1-7-0	30.3	281.25	3	56.25	86.65
	0-6-5-9-0	17.7	279.90		55.98	
	0-4-3-8-10–0	65.3	332.15		66.43	

**Table 9:** Distribution costs under cooperation between Yunda and Zhongtong

Zhongtong-Yunda joint distribution	Distribution route	Mileage	Traffic demand	Transfer vehicle	Loading rate (%)	Distribution cost
Yunda	0-5-4-6-2-9-0	37.4	895.94	2	89.59	38.7
Zhongtong	0-7-1-3-8-10-0	68.7	924.69	2	92.47	54.35
Yuantong	0-4-2-6-9-0	42.2	423.30	3	84.66	103.7
	0-7-1-0	40.5	179.31		35.86	
	0-5-3-8-10–0	64.7	441.70		88.34	

**Table 10:** Distribution costs under the cooperation of three enterprises.

Joint distribution by three enterprises	Distribution route	Mileage	Traffic demand	Transfer vehicle	Loading rate (%)	Distribution cost
Yuantong	0-4-5-6-0	33.9	912.48	1	91.25	36.95
Zhongtong	0-2-1-7-9-0	29.9	998.35	1	99.83	34.95
Yunda	0-3-8-10-0	35.8	954.11	1	95.41	37.9

**Table 11:** Organizational benefits under various modes of cooperation.

Distribution plan	Total distribution cost	Revenue from joint distribution
Three separate distributions	285.95	0
Joint distribution between enterprises 1 and 2	194.85	91.1
Joint distribution between enterprises 1 and 3	179.8	106.15
Joint distribution between enterprises 2 and 3	196.75	89.2
Three joint distributions	109.8	176.15

**Table 12:** Calculation table of the initial Shapley value of the Yuantong enterprise.

*S*	{1}	{1, 2}	{1, 3}	{1, 2, 3}
*V*(*S*)	0	91.1	106.15	176.15
*V*(*S* − {1})	0	0	0	89.2
*V*(*S*) − *V*(*S* − {1})	0	91.1	106.15	86.95
|*S*|	1	2	2	3
*ω*(*S*)	1/3	1/6	1/6	1/3
*ω*(*S*)[*V*(*S*) − *V*(*S* − {*i*})]	0.00	15.19	017.70	29.98

**Table 13:** Calculation table of the initial Shapley value of the Zhongtong enterprise.

*S*	{2}	{2, 1}	{2, 3}	{1, 2, 3}
*V*(*S*)	0	91.1	89.2	176.15
*V*(*S* − {2})	0	0	0	106.15
*V*(*S*) − *V*(*S* − {2})	0	91.1	89.2	70
|*S*|	1	2	2	3
*ω*(*S*)	1/3	1/6	1/6	1/3
*ω*(*S*)[*V*(*S*) − *V*(*S* − {*i*})]	0.00	15.19	14.87	23.33

**Table 14:** Calculation table of the initial Shapley value of the Yunda enterprise.

*S*	{3}	{3, 1}	{3, 2}	{1, 2, 3}
*V*(*S*)	0	106.15	89.2	176.15
*V*(*S* − {3})	0	0	0	91.1
*V*(*S*) − *V*(*S* − {3})	0	106.15	89.2	85.05
|*S*|	1	2	2	3
*ω*(*S*)	1/3	1/6	1/6	1/3
*ω*(*S*)[*V*(*S*) − *V*(*S* − {*i*})]	0.00	17.70	14.87	28.35

**Table 15:** Correction factors of enterprises from the perspective of groups.

Cooperation mode of shared resources	Weight	Enterprise 1	Enterprise 2	Enterprise 3
Strength and status of the members of the alliance	0.5	0.53	0.32	−0.85
Service unit price and market demand	0.3	0.83	0.76	−1.59
Stability of logistics alliance	0.2	−0.43	0.26	0.17
Correction factor of enterprise i	—	0.43	0.44	−0.87

**Table 16:** Correction factors of each enterprise from an individual perspective.

Coordination mechanism of income distribution	Weight	Enterprise 1	Enterprise 2	Enterprise 3
Cost input	0.3	0.54	0.34	−0.88
Risk bearing	0.3	0.36	0.27	−0.63
Service level	0.3	0.47	0.37	−0.84
Marginal contribution	0.1	0.31	0.29	−0.6
Correction factor of enterprise i	—	0.44	0.32	−0.77

**Table 17:** Corrections for each enterprise.

	Yuantong	Zhongtong	Yunda
Correction factor	0.31	0.24	−0.55
Correction value	18.90	12.95	−33.38

**Table 18:** Comparison of results before and after correction.

	Yuantong	Zhongtong	Yunda
Shapley value method	61.86	53.39	60.91
After correction	18.90	12.95	−33.38

## Data Availability

The data generated and analyzed during this research are available from the corresponding author on request.
